The article "Observation on the Effect of Solution-Focused Approach Combined with Family Involvement in WeChat Platform Management on Inpatients with Intracerebral Hemorrhage" was published in 2022. Journal: J Healthc Eng.

# Observation on the Effect of Solution-Focused Approach Combined with Family Involvement in WeChat Platform Management on Inpatients with Intracerebral Hemorrhage

**DOI:** 10.1155/2022/9951374

**Published:** 2022-03-19

**Authors:** Yu Song

**Affiliations:** Department of Neurology, The First Affiliated Hospital of Harbin Medical University, Harbin 150001, Heilongjiang Province, China

## Abstract

**Objective:**

To explore the effect of the solution-focused approach combined with family involvement in the WeChat platform management on inpatients with intracerebral hemorrhage (ICH).

**Methods:**

A total of 80 ICH patients hospitalized in our hospital from June 2018 to June 2021 were split into the control group (CG) and the study group (SG) according to the clinical nursing modes, with 40 cases in each group. Both groups received routine intervention, while SG additionally received the solution-focused approach combined with family involvement in the WeChat platform management to compare the self-care ability, psychological status, and hope levels between the two groups after intervention.

**Results:**

No significant differences in general data were observed between the two groups (*P* > 0.05). The SAS and SDS scores before intervention showed mild depression and anxiety in both groups, which improved after intervention. In addition, the SAS and SDS scores after intervention were remarkably lower in SG than in CG (*P* < 0.05). After intervention, the scores of ICH-related knowledge, self-care skills, self-care responsibility, and rehabilitation knowledge in SG were notably higher compared with CG (*P* < 0.05). After intervention, the Herth scores of both groups increased, with a higher score in SG than in CG (*P* < 0.05). After intervention, SG had higher quality of life (QOL) scores in general health, physiological function, physiological role, body pain, vitality, social function, emotional role, and physiological health than CG (*P* < 0.05).

**Conclusion:**

The implementation of the solution-focused approach combined with family involvement in the WeChat platform management for ICH inpatients can effectively improve their psychological status, enhance their self-care ability and hope levels, promote body recovery, and improve their QOL after intervention.

## 1. Introduction

Intracerebral hemorrhage (ICH) is a common clinical disease with an urgent onset, which is mainly related to cerebrovascular diseases such as hyperlipidemia, diabetes, hypertension, and vascular aging. With a high early mortality rate, patients often suffer from a sudden onset due to emotional excitement and hard work, and most survivors experience various sequelae such as cognitive impairment, motor impairment, and language disorders. Faced with the stress of sudden onset, unpredictability, and long-term rehabilitation of the disease, patients often show psychological stress reactions such as anxiety and depression, affecting the rehabilitation and even aggravating the disease [1–4]. Therefore, it is necessary to explore an intervention method that can improve the physical and mental status of ICH patients. The solution-focused approach is a new nursing intervention model in clinical practice in recent years with the core purpose of exploring solutions to solve problems and the purpose of improving the adverse status of patients through positive, goal-oriented, and problem-solving perspectives, which may have a positive impact on ICH inpatients [5–8]. Besides, clinical practice has found that ICH patients are accompanied by a long-term recovery process, and their lifestyle, medication compliance, and physical exercise habits after intervention directly affect the physical rehabilitation effect of patients. Based on this, our hospital intervened ICH inpatients through the solution-focused approach to improve their adverse status and ensure the rehabilitation effect. In addition, family involvement in the WeChat platform management was performed to further guarantee the effectiveness of clinical intervention and improve the quality of life (QOL) of patients after intervention. At present, there are few related studies. In this study, 80 ICH patients in our hospital were selected as the research subjects, which is further discussed in this study.

## 2. Study Protocol

### 2.1. Case Screening

Eighty ICH patients hospitalized in our hospital from June 2018 to June 2021 were split into the control group (CG) and the study group (SG) according to the clinical nursing modes, with 40 cases in each group. Both groups received routine intervention, while SG additionally received the solution-focused approach combined with family involvement in the WeChat platform management. The study obtained the approval and supervision of the hospital ethics committee.

### 2.2. Inclusion Criteria

The inclusion criteria were as follows: (1) patients met the clinical diagnostic criteria of ICH [9] and were confirmed by imaging data of MRI and CT; (2) patients had a systolic pressure of no more than 140 mmHg or a diastolic pressure of no less than 90 mmHg (stable blood pressure levels); (3) patients had no cognitive or communication barriers; (4) patients had family members who accompanied them for a long time and were skilled in WeChat function; (5) patients had the first onset; and (6) patients and their families were informed of and agreed to this study.

### 2.3. Exclusion Criteria

The exclusion criteria were as follows: (1) patients with severe organ dysfunction or malignant tumors; (2) patients with extremely unstable basic indicators such as blood pressure, blood glucose, and blood lipid; (3) patients with poor cooperation or discharged halfway; (4) patients with incomplete clinical data; (5) patients with intracranial infection; and (6) patients with unclear consciousness, visual or auditory impairment, and language barriers.

## 3. Methods

Routine intervention was performed as discussed further. The nursing staff paid attention to the patients' changes in vital signs, consciousness, and condition, evaluated their language competence, limb activity, and pupil changes, understood their degree of neurological impairment, and paid attention to their respiratory management and medication according to the doctor's advice. The staff also paid attention to the psychological changes of patients, timely implemented psychological intervention, improved the awareness of patients and their families on the disease through effective health education, and helped them concentrate on the clinical treatment and rehabilitation training. While ensuring the nursing quality, nurses encouraged patients with similar conditions to communicate with each other to reduce loneliness and anxiety caused by the disease and enhance their confidence in the body rehabilitation [10–12]. Targeted rehabilitation programs were developed such as active activities of joints and limbs, and position changing to strengthen the patients' activities of daily living and physiological function exercise. According to the principle of gradual treatment, individualized scientific and effective rehabilitation training should be implemented, with the amount of rehabilitation training ranging from small to large. The training content was dominated by single functional training such as motor and sensation and gradually transitioned to the improvement of activities of daily living.

The solution-focused approach combined with family involvement in the WeChat platform management was implemented as follows. First, after an intervention group of a solution-focused approach was established, all-round training on ICH rehabilitation knowledge and a solution-focused approach was carried out, and the nursing process was divided into describing problems, building specific and feasible goals, exploring exceptions, providing feedback, and evaluating the progress. (1) Describing problems: after admission of the patients, the staff had a detailed understanding of their general information, informed them and their families of possible problems during the rehabilitation process, and provided feasible solutions to the problems, thus increasing patients' confidence in rehabilitation. (2) Building specific and feasible goals: the staff understood the family situation and rehabilitation needs of patients and their families through in-depth conversation with them, developed feasible rehabilitation goals, and formulated comprehensive exercise programs together with the patients and families, providing scientific guidance and seeking family cooperation [13, 14]. (3) Exploring and solving problems: by sharing previous successful rehabilitation cases with patients, the staff encouraged them to face the rehabilitation process with a positive attitude and knew their psychological changes and treatment experiences through lectures, communication between patients, and one-on-one conversation. (4) Feedback: the staff regularly discussed the patients' progress of rehabilitation training, summarized their advantages and body function changes, timely adjusted goals and programs, and gave the patients positive feedback in the way of language encouragement and praise, so as to improve their treatment enthusiasm and encourage them to work towards the preset goals. For the patients with unsatisfactory rehabilitation effects, the staff encouraged them, objectively analyzed the reasons, and tried other effective rehabilitation measures to support them. (5) Evaluation of the progress: the staff evaluated the symptoms, signs, psychological status, and recovery of patients, summarized the experience, set new rehabilitation goals according to the changes in the condition and the needs of patients, refined the overall goals, reflected the patients' progress in a more intuitive way, and improved their confidence in working towards the next goal. The WeChat platform management with family involvement was detailed as follows. On the basis of routine intervention, a special WeChat group was set up for each patient to form a management platform composed of doctors, nurses, and family members of patients, and intervention was carried out through this platform. (1) The WeChat management platform was established by the intervention group using a solution-focused approach, involving 1–2 family members for each patient. (2) The members of the management group regularly pushed ICH-related health knowledge to the family members through the WeChat platform, such as diagnosis, treatment, nursing, and prevention of ICH [15]. (3) Through the WeChat platform, the medical staff timely answered the questions of patients and their families, conducted disease analysis, and adjusted treatment plans. (4) For patients with hyperemia, family members of patients should regularly upload the blood pressure levels and medication of patients. (5) All patients were notified through the WeChat platform for regular reexamination and adjustment of the medication schemes, and follow-up was performed after intervention.

### 3.1. Observation Indexes

1. The age, BMI, blood loss, gender, bleeding sites, bleeding causes, and education level of the patients were recorded at admission.
2. Psychological status. The *Self-rating Anxiety Scale (SAS)* and the *Self-rating Depression Scale (SDS)* were used to evaluate the psychological status of patients. According to the Chinese norms, a SAS score below 50 points represented a normal state, with 50–59 as mild anxiety, 60–69 as moderate anxiety, and a score of no less than 70 as severe anxiety. An SDS score below 53 points represented normal state, with 53–62 as mild depression, 63–72 as moderate depression, and a score of more than 72 as severe depression.
3. Self-care ability. The *Self-Care Ability Assessment Scale* adapted by Zia et al. [16] was adopted to assess the self-care ability of ICH patients, including four dimensions of ICH-related knowledge, self-care skills, self-care responsibility, and rehabilitation knowledge, each scoring 100 points. Higher scores suggest a stronger self-care ability of the patients.
4. Hope levels. The *Herth Hope Scale* was used to evaluate the hope levels of ICH patients, including a positive attitude towards reality and the future, positive action, and maintaining close relations with others, with a total of 12 items. Each item was scored according to the four-level scoring method (1–4 points), and the total score was divided into three levels: low level (12–23 points), medium level (24–35 points), and high level (36–48 points). This scale had a Cronbach's *α* of 0.971, with good reliability and validity.
5. QOL. The patients were assessed using the SF-36 scale, including general health, physiological function, physiological role, body pain, vitality, social function, emotional role, and physiological health. The reliability coefficient of each dimension was 0.721–0.869, with good reliability and validity. Higher scores suggested better QOL of the patients.

### 3.2. Statistical Treatment

The data were calculated by the software SPSS22.0 and graphed by GraphPad Prism 7 (GraphPad Software, San Diego, USA). The data included enumeration and measurement data, expressed as (*n* (%)) and (‾*x* ± *s*) and tested by X^2^ and *t*-test. When *P* < 0.05, the differences were statistically significant.

## 4. Results

### 4.1. General Information

No statistical differences in age, BMI, blood loss, gender, bleeding sites, bleeding causes, and education levels were observed between the two groups (*P* > 0.05), as shown in Table 1.

### 4.2. Psychological Status

The SAS and SDS scores before intervention showed mild depression and anxiety in both groups, which improved after intervention. In addition, the SAS and SDS scores after intervention were remarkably lower in SG than in CG (*P* < 0.05), as presented in Table 2.

### 4.3. Self-Care Ability

After intervention, the scores of ICH-related knowledge, self-care skills, self-care responsibility, and rehabilitation knowledge in SG were notably higher compared with CG (*P* < 0.05), as shown in Figure 1.

### 4.4. Hope Levels

After intervention, the Herth scores of both groups increased, with a higher Herth score in SG than in CG (*P* < 0.05), as presented in Figure 2.

The Herth scores in SG before and after intervention were (24.50 ± 4.07) and (36.15 ± 3.37). ^*∗*^represents a notable difference in the Herth scores between the two groups after intervention (*t* = 8.756, *P* < 0.001).

### 4.5. QOL

After intervention, SG had higher QOL scores in general health, physiological function, physiological role, body pain, vitality, social function, emotional role, and physiological health than CG (*P* < 0.05), as shown in Table 3.

## 5. Discussion

The solution-focused approach is an intervention model of clinical central psychotherapy, which has gradually developed into an intervention model in nursing rehabilitation after clinical practice [17–20]. This model respects individuals and improves patients' subjective initiative during rehabilitation by constantly tapping into their own resources and potential. By focusing on solving the problems, it makes up for the deficiencies of the traditional model that blindly instills functional exercise knowledge into patients, and pays more attention to stimulating their application and coping ability, thus enhancing their initiative and participation, and being more easily accepted by patients [21–24]. Compared with the traditional problem-solving model, the solution-focused approach is a clinical intervention model developed on the background of positive psychology that fully respects individuals and believes in their own resources and potential. It emphasizes the focus of problem-solving on the positive aspects of people and the maximization of the strengths, advantages, and capabilities of individuals or groups. This model believes that it is unnecessary to explore the causes in order to promote the occurrence of changes, which is in great contrast to the traditional problem-solving model that explores the causes of problems and leads to solutions. At present, this model is widely used in clinical psychological intervention. At present, effective health education is also the key to ensuring the clinical efficacy of patients. For ICH patients, maintaining a good attitude, a healthy lifestyle and diet, and regular reexamination are the keys to affecting the efficacy after intervention. To ensure that patients maintain a good attitude and healthy living habits throughout the long rehabilitation process, our hospital implemented the WeChat platform management with family involvement for ICH patients, and its combined intervention with the solution-focused approach remarkably improved the QOL of patients after intervention.

After the onset of the disease, patients are prone to negative emotions such as anxiety and depression due to the lack of living ability, long recovery period, and huge psychological pressure. Through the implementation of the solution-focused approach combined with family involvement in the WeChat platform management, this study tried to solve the patients' mental health problems. It was concluded that the SAS and SDS scores before intervention showed mild depression and anxiety in both groups, which improved after intervention. In addition, the SAS and SDS scores after intervention were remarkably lower in SG than in CG (*P* < 0.05). These were in line with the study by Maureen Chila [25], confirming that the solution-focused approach guides patients to solve their own problems. By establishing the goals to stimulate the potential, the approach helps the patients clarify the problems and explore solutions to complete the established and feasible goals, thereby improving their confidence in overcoming the disease. At present, drugs are often used to control the negative emotions of patients in clinical practice, supplemented by traditional psychological intervention. However, due to various subjective factors affecting emotions, drug therapy is difficult to solve the fundamental problems. The solution-focused approach combined with family involvement in the WeChat platform management helps patients solve problems such as bad lifestyle and eating habits, and insomnia. At the same time, close attention from relatives also increases the confidence of patients and promotes the elimination of negative emotions. After intervention, the scores of ICH-related knowledge, self-care skills, self-care responsibility, and rehabilitation knowledge in SG were notably higher compared with CG (*P* < 0.05). The Herth scores of both groups increased after intervention, with a higher Herth score in SG than in CG (*P* < 0.05). The results confirm that solving the problems is the key link in the rehabilitation and treatment of patients. The solution-focused approach improves the psychological status of patients, focuses on solving the practical problems and potential mining of patients, stimulates active participation, enhances self-management ability, and boosts psychological resilience and hope levels. The intervention of the WeChat platform has promoted a close relationship between doctors and patients, and between patients and their families, and improved the patients' treatment compliance with the support from multiple aspects. At the same time, this model further strengthens the supervision and reminding of patients. Finally, SG had higher quality of life scores in general health, physiological function, physiological role, body pain, vitality, social function, emotional role, and physiological health than CG after intervention (*P* < 0.05), showing the combined intervention can fundamentally improve the QOL of patients. This research was a single-center study with a small sample size, in which only 80 patients were statistically analyzed. In the subsequent studies, the sample size needs to be expanded to further confirm the intervention effect of the solution-focused approach combined with family involvement in the WeChat platform management on the ICH patients. As for the solution-focused approach in practice, the patients' habitual thinking tends to hinder the new way of thinking. For example, the patients may restore their original thinking after intervention, which requires the intervener to continuously obtain the recognition of the patients in the implementation process and increase the intervention frequency. With considerable overall effect, the WeChat platform management does not intervene the patients directly, such as the education of early nursing mainly on the family members of patients. Therefore, attention should be paid to the efficiency of the family members on the platform in practice.

In conclusion, the implementation of the solution-focused approach combined with family involvement in the WeChat platform management for ICH inpatients can effectively improve their psychological status, enhance their self-care ability and hope levels, promote body recovery, and improve their QOL after intervention.

## Figures and Tables

**Figure 1:** Comparison of self-care ability after intervention. Note: the abscissa represented the evaluation dimensions, and the ordinate represented the score (points). The scores of ICH-related knowledge, self-care skills, self-care responsibility, and rehabilitation knowledge in CG were (80.40 ± 9.91), (77.62 ± 10.85), (77.29 ± 10.51), and (78.03 ± 10.53), respectively. The scores of ICH-related knowledge, self-care skills, self-care responsibility, and rehabilitation knowledge in SG were (89.64 ± 9.75), (88.45 ± 9.72), (87.52 ± 10.50), and (90.12 ± 9.43), respectively. ^*∗*^indicates notable differences in the scores of ICH-related knowledge, self-care skills, self-care responsibility, and rehabilitation knowledge between SG and CG (*t* = 4.204, 4.702, 4.355, 5.409; *P* < 0.05).

**Figure 2:** Comparison of Herth scores. Note: the abscissa represents before and after intervention, and the ordinate represents the score (points). The Herth scores in CG before and after intervention were (24.33 ± 4.20) and (30.04 ± 2.85). The Herth scores in SG before and after intervention were (24.50 ± 4.07) and (36.15 ± 3.37). ^∗^represented a notable difference in the Herth scores between the two groups after intervention (t = 8.756, P < 0.001).

**Table 1:** Comparison of general data.

Observation indexes	CG	SG	X^2^/*t*	*P*
Age (years)	58.22 ± 7.18	58.47 ± 7.15	0.156	0.876
BMI (kg/m^2^)	23.59 ± 3.11	23.52 ± 3.10	0.101	0.920
Blood loss (ml)	16.72 ± 5.44	16.43 ± 5.51	0.237	0.813
Gender (male/female)	28/12	27/13	0.058	0.809
Bleeding sites				
Basal ganglia	25 (62.5)	23 (57.5)	0.208	0.648
Thalamus	7 (17.5)	9 (22.5)	0.313	0.576
Ventricles	4 (10)	5 (12.5)	0.125	0.723
Cerebral lobes	4 (10)	3 (7.5)	0.157	0.692
Bleeding causes				
Hypertension	26 (65)	25 (62.5)	0.054	0.816
Arteriolosclerosis	10 (25)	9 (22.5)	0.069	0.793
Others	4 (10)	6 (15)	0.457	0.499
Education levels			0.474	0.491
Junior high school and below	23 (57.5)	26 (65)		
Above junior high school	17 (42.5)	14 (35)		

**Table 2:** Comparison of SAS and SDS scores.

Indexes		CG	SG	t/*P*
SAS	Before intervention	61.18 ± 6.71	61.34 ± 6.50	
	After intervention	52.05 ± 5.81^*∗*^	48.32 ± 4.67^*∗*^	3.141/0.002
SDS	Before intervention	56.43 ± 4.26	56.81 ± 4.19	
	After intervention	53.61 ± 3.15^*∗*^	46.05 ± 3.11^*∗*^	10.801/<0.001

Note: ^*∗*^*P* < 0.05, compared with that before intervention within the same group.

**Table 3:** Comparison of SF-36 scores.

Evaluation dimensions	CG	SG	t	*P*
General health	80.62 ± 9.47	91.17 ± 6.55	5.795	<0.001
Physiological function	80.55 ± 8.73	90.08 ± 7.41	5.264	<0.001
Physiological role	78.29 ± 7.40	87.02 ± 7.11	5.380	<0.001
Body pain	79.04 ± 8.27	90.04 ± 7.80	6.120	<0.001
Vitality	79.35 ± 9.83	88.29 ± 7.15	4.652	<0.001
Social function	76.50 ± 8.55	90.01 ± 7.70	7.426	<0.001
Emotional role	77.09 ± 8.25	88.47 ± 8.11	6.221	<0.001
Physiological health	77.34 ± 8.86	89.35 ± 9.13	5.970	<0.001

## Data Availability

The data supporting the findings of this study are available from the corresponding author on reasonable request.
